This article has been retracted.

# National income accounting attributes and economic welfare. Evidence from Pakistan

**DOI:** 10.1371/journal.pone.0301829

**Published:** 2024-08-08

**Authors:** Yang Shuang, Muhammad Waris, Muhammad Kashif Nawaz, Cheng Chan, Ijaz Younis

**Affiliations:** 1 Xinyang Vocational and Technical College, Henan, Xinyang, China; 2 School of Business, University of Education Multan Campus, Multan, Pakistan; 3 Institute of Management Sciences, Bahauddin Zakariya University, Multan, Pakistan; 4 School of management, Guangzhou University, Guangzhou, PR China; National University of Modern Languages, PAKISTAN

## Abstract

Economic welfare is essential in the modern economy since it directly reflects the standard of living, distribution of resources, and general social satisfaction, which influences individual and social well-being. This study aims to explore the relationship between national income accounting different attributes and the economic welfare in Pakistan. However, this study used data from 1950 to 2022, and data was downloaded from the World Bank data portal. Regression analysis is used to investigate the relationship between them and is very effective in measuring the relationship between endogenous and exogenous variables. Moreover, generalized methods of movement (GMM) are used as the robustness of the regression. Our results show that foreign direct investment outflow, Gross domestic product growth rate, GDP per capita, higher Interest, market capitalization, and population growth have a significant negative on the unemployment rate, indicating the rise in these factors leads to a decrease in the employment rate in Pakistan. Trade and savings have a significant positive impact on the unemployment rate, indicating the rise in these factors leads to an increase in the unemployment rate for various reasons. Moreover, all the factors of national income accounting have a significant positive relationship with life expectancy, indicating that an increase in these factors leads to an increase in economic welfare and life expectancy due to better health facilities, many resources, and correct economic policies. However, foreign direct investment, inflation rate, lending interest rate, and population growth have significant positive effects on age dependency, indicating these factors increase the age dependency. Moreover, GDP growth and GDP per capita negatively impact age dependency. Similarly, all the national income accounting factors have a significant negative relationship with legal rights that leads to decreased legal rights. Moreover, due to better health facilities and health planning, there is a negative significant relationship between national income accounting attributes and motility rate among children. Our study advocated the implications for the policymakers and the government to make policies for the welfare and increase the social factors.

## Introduction

With rapid expansion, industrial innovation, and changing economic landscapes, emerging economies provide a fascinating area for studying national income accounting and its substantial consequences for economic well-being. Traditional economic performance indicators, such as Gross Domestic Product (GDP), generally show a picture of success and expansion in these countries [1]. However, this picture merely touches the surface of the intricate relationship between economic progress and population well-being. As we go deeper into this issue, it becomes clear that knowing the characteristics of national income accounting and their direct impact on economic welfare is critical nationally and globally [2, 3]. Emerging economies face many problems as they seek greater prosperity [4]. While national accounting attributes are frequently highlighted, it is equally vital to assess how this economic expansion translates into actual improvements in the quality of life for their population. Income inequality, resource allocation, job creation, environmental sustainability, and social development are essential elements that must be considered when evaluating economic welfare [5].

Indeed, economic welfare is a fascinating topic of study, with continuous challenges and questions that attract economists, politicians, and scholars. However, the global economic welfare problem refers to the challenges and issues related to people’s well-being and economic prosperity worldwide. Several critical economic welfare problems are prevalent on a global scale. Unemployment remains a significant challenge in many parts of the world [6]. The International Labor Organization estimated that the global youth unemployment rate would be 13.1% in 2021, and the global working poverty rate would be 9.0% (ILO, 2021). This results in reduced incomes, limited access to education and healthcare, and lower living standards, impacting economic welfare.

Moreover, unemployment is a persistent and fascinating academic topic, particularly in rising and developing nations [7]. It is a multidimensional problem with significant economic, social, and political ramifications. A large number of the studies focus on the structural nature of unemployment in emerging economies. Unemployment is caused by a mismatch between the skills of the labor force and the abilities required by businesses [8]. This problem is exacerbated by educational gaps, a lack of vocational training programs, and changing industrial requirements (World Bank, 2019).

Access to quality education and healthcare is crucial for economic welfare [9]. Disparities in access to education and healthcare services persist globally, with many individuals and communities facing limited opportunities for skill development and reduced productivity (World Bank, 2018). Legal rights such as protectionism, trade disputes, and uneven trade agreements can result in economic imbalances, reduced market access, and hindered economic growth [10]. Inadequate regulation and governance of financial systems can also lead to financial crises and economic instability, impacting global economic welfare [11]. Demographic challenges, such as aging populations, migration, and rapid urbanization, can also impact global economic welfare. Aging populations in many countries can strain social welfare systems, reduce the labor force, and affect economic growth (Bloom et al., 2021).

However, the unemployment rate remains challenging for every global economy [12]. Every economy wants to balance the unemployment rate to stabilize economic indicators [13]. This task may be worsened or accessible with the balanced national income accounting attributes that create an exciting gap for investigation. However, it is interesting to investigate the influence of the national income attributes on the unemployment rate in emerging economies.

Moreover, life expectancy and age dependency are also exciting challenges to the economy in providing health facilities to their citizens, especially in emerging economies with a lack of economic resources [14]. However, this study will investigate the influence of the national income attributes on life expectancy and age dependency in emerging economies that have gotten little attention. Legal rights are integral to citizenship in both emerging and established countries [15]. Legal rights comprise various individual rights and protections in a country’s legal system [16]. These rights ensure that citizens are treated fairly, justly, and with dignity following the law. However, it is interesting to investigate the influence of the national income attributes on the legal rights in emerging economies.

Moreover, the mortality rate in children is worth much attention now because of the shortage of nutrition facilities in the emerging economy [17]. However, there are limited studies on the mortality rate and the national income attributes, especially in emerging economies. Moreover, this study aims to explore the work of the Gibbons, Sprong [18].

The gross savings rate in Pakistan is updated annually, containing data from June 2000 to June 2023, with an average rate of 6.0%. Notably, the data peaked at 6.0% in June 2003 and reached a low of 3.8% in June 2022 [19]. GDP per capita in Pakistan will average $1474 in 2023, which is expected to rise in 2024 [19]. Moreover, in November 2023, Pakistan had a significant increase in foreign direct investment (FDI), totaling 131.4 million USD [19]. This contrasts with the previous month’s growth, which totaled 122.5 USD million. In 2023, Pakistan’s Stock market capitalization was $27 Billion [19]. In September 2023, Pakistan’s annual inflation rate reached a four-month high of 31.4%, up from 27.4% the previous month. The primary reason for this increase is fuel and energy prices. The population growth rate in Pakistan was 1.98% in 2023 [19]. Moreover, the unemployment rate will peak in 2023, reaching 8.5%. Life expectancy increased by 0.21% from the previous year. The mortality rate in newborn children is higher than 6.7% in 2023. Fig 1 shows the current state.

**Fig 1:** Current statistics about national income accounting and economic welfare.

Our findings contribute to the existing literature by providing fresh evidence related to the economic welfare of the emerging economy, especially Pakistan. Moreover, it contributed to the body of knowledge in the literature that the negative impact of FDI outflow on unemployment suggests that when Pakistani firms invest abroad, it may reduce employment opportunities in the domestic market. On the other hand, the positive impact of FDI inflow on reducing unemployment implies that foreign investments in Pakistan may create jobs and contribute to employment opportunities in the local economy.

However, it also added to the previous literature the negative impact of GDP and GDP per capita on unemployment, indicating that higher levels of economic growth are associated with lower unemployment rates in Pakistan. This supports the notion that economic growth can contribute to increased employment opportunities and emphasizes the importance of policies that promote GDP growth for addressing unemployment challenges in Pakistan. Similarly, it highlights the role of interest rates in shaping unemployment trends.

The negative impact of interest rates on unemployment suggests that higher interest rates may hinder employment opportunities in Pakistan. This finding underscores the importance of monetary policies maintaining stable interest and inflation rates for promoting employment generation. Another contribution to the body of knowledge is the positive impact of trade and savings on unemployment, indicating that higher trade and savings may contribute to lower unemployment rates in Pakistan. This finding suggests that policies promoting international trade and encouraging savings can play a crucial role in addressing unemployment challenges in the country.

Moreover, the study provides insights into the impact of national income accounting factors, such as GDP, GDP per capita, and interest rates, on age dependency. The adverse effects of these factors on age dependency suggest that higher economic growth and lower interest rates may lead to a decrease in the dependency ratio, which is the proportion of dependent individuals (typically children and elderly) relative to the working-age population. This finding highlights the potential of economic growth and favorable interest rate policies in reducing the burden of age dependency on the working-age population in Pakistan. Sixthly, the study suggests that FDI, savings, and trade positively impact age dependency, indicating that these factors may contribute to an increase in the dependency ratio. This finding underscores the need to consider the potential demographic implications of policies related to FDI, savings, and trade in Pakistan. Lastly, the study reveals that national income accounting factors have a negative impact on legal rights but a positive impact on reducing child mortality rates in Pakistan. This finding suggests that higher national income levels may be associated with improved access to education, health care, and social services, leading to overall socio-economic development and reduced child mortality rates. However, the negative impact on legal rights suggests that there may be trade-offs between economic development and legal rights. It underscores the need for policies that balance economic growth with social and legal protections. Moreover, our study advocated the implications for policymakers, practitioners, and other stakeholders.

The remaining sections of this article are structured as follows: Part 2 presents an overview of recent literature and theoretical background and puts forward several hypotheses that can be tested to understand the relationship between variables better. The conceptual framework, research design, and methods are detailed in Part 3. Part 4 outlines the study’s findings, while Part 5 encompasses the conclusion, suggestions for further research, limitations, and practical implications.

### Literature review and theoretical background

Several theories support studying the relationship between national income accounting and economic welfare. These theories provide insights into the complex dynamics and factors that influence economic welfare and emphasize the need for a multidimensional approach to assessing economic welfare beyond traditional national income accounting measures. Amartya Sen’s capability approach argues that economic welfare should be measured in terms of individuals’ capabilities and freedoms to live fulfilling lives [20]. Sen argues that traditional income measures, such as GDP, do not capture the diverse capabilities and freedoms that individuals need to achieve well-being [21]. Moreover, this theory emphasizes the importance of education, health, and social opportunities in determining economic welfare. Sen’s capability approach highlights the need to consider a range of dimensions beyond income in assessing economic welfare. It aligns with the call for a multidimensional approach to national income accounting [21].

The sustainable development theory emphasizes the need to account for environmental sustainability in assessments of economic welfare. It argues that economic development should not come at the cost of environmental degradation and have negative consequences for future generations. Moreover, the theory emphasizes the importance of incorporating environmental indicators, such as natural resource depletion, pollution, and climate change impacts, in national income accounting frameworks to ensure sustainable economic welfare for present and future generations (World Commission on Environment and Development, 1987).

According to Mitchell, Weaver [22], the social welfare function theory argues that economic welfare should be evaluated based on social preferences and values. Moreover, it highlights the subjective nature of economic welfare and the importance of incorporating societal preferences in assessing well-being. It emphasizes the need for participatory approaches and stakeholder engagement in national income accounting to ensure that different groups’ diverse needs and preferences are considered [22].

According to Silva, Goosby [23], life expectancy has decreased due to the COVID-19 case in the U.S. They also concluded that more investment is needed for economic welfare. However, Barbier and Burgess [24] concluded that long-term improvement should be required to increase economic welfare’s average age and life expectancy. These theories provide theoretical foundations and frameworks that support the study of the relationship between national income accounting and economic welfare. Most theories emphasize the need to go beyond traditional income measures and incorporate a multidimensional approach to assessing economic welfare, considering human development, environmental sustainability, income distribution, and societal preferences. Combining these theories provides a road map to understand the relationship of the problems taken as study.

According to Gutter and Copur [25], higher levels of national savings contribute positively to economic welfare by increasing life expectancy, reducing the unemployment rate, achieving legal rights, and decreasing the mortality rate in children due to food scarcity. According to Aizenman and Sengupta [26], countries with higher savings rates tend to invest more in physical and human capital, promoting economic growth and development. National income accounting, which involves measuring and analyzing a country’s economic performance, has been widely used to assess economic welfare.

Previous literature has shed light on the strengths and limitations of using national income measures as welfare indicators. Still, there is a gap in the literature to investigate most measures of national income accounting and economic welfare. One of the critical concepts in national income accounting is Gross Domestic Product (GDP), which measures the total value of goods and services produced within a country’s borders during a specific period [27]. GDP is often used as a proxy for economic welfare, as higher GDP is assumed to reflect higher levels of economic activity and well-being [28]. However, there are limitations to using GDP as the sole indicator of economic welfare.

Various studies such as Stiglitz [29], MacFeely and van de Ven [30] have shown that GDP may not fully capture the well-being of a population, as it does not account for factors such as income distribution, environmental sustainability, and social indicators such as education, health, and happiness. According to Ren, Guo [31], a country with high GDP may still have significant income inequality, environmental degradation, and low levels of social welfare, which negatively impact overall economic welfare. According to Eldeep and Zaki [32], relying solely on GDP to assess economic welfare may result in an incomplete picture. Still, there is a need for similar factors that impact economic welfare together with GDP.

According to Nazif and Jenkins [33], savings have greatly contributed to the gross domestic product and significantly impacted economic welfare by reducing the rate of unemployment among youth and old persons. Moreover, Peprah, Peprah [34] defined that some social and economic factors contributed to increasing economic welfare. Furthermore, these benefits were visible in categories such as income, contribution to household expenditure, home decision-making, community engagement, family nutrition, access to education for wards, asset acquisition, and quality housing.

According to van der Heide and Kohl [35], market capitalization increases life expectancy through insurance and other factors that contribute significantly towards economic welfare. Moreover, Jha and Kelley [36] stated that social networks are also related to much better probabilities of a household favorably perceiving its financial status. Social capital multiplies household well-being across various dimensions [37].

Jerneck [38] stated that economic policy is structured by the notion that tax money is scarce and that the state should keep a balanced budget. According to Römer [39], increased immigration spending is projected to come at the expense of the welfare state. Each immigrant is regarded to impose a cost on society until they can find work. In the meantime, the austere fiscal policy limits employment levels. As a result, anti-immigrant sentiments and calls for welfare are on the rise.

However, according to Dosis [40], low-interest rates and a lack of entrepreneurial wealth allow unproductive businesses to enter the pool of borrowers. Due to this knowledge externality, profit enterprises are forced to reduce their investment levels. In some circumstances, interest rate rises have equivocal effects on total investment and production while increasing economic welfare. According to Ikotun, Ezugwu [41], economic development includes GDP and yearly foreign direct investment, which have a considerable negative impact on human well-being.

Nonetheless, this influence is erratic, indicating that these countries should choose sustainable development strategies cautiously. Similarly, Dempere, Qamar [42] investigated that innovation has a favorable impact on human resources, research, and creative outputs but has little effect on FDI. According to the findings, a workable regulatory framework, institutional support, domestic human resources, research and development, infrastructure, technology, and creative outputs are all necessary for a thriving economy. According to Wirajing, Nchofoung [43] that there is inequality is found due to the high population growth that leads to a decrease in economic welfare due to a lack of resources in the country, and these types of problems faced by lower as well as middle-income countries.

According to Hongming, Ahmed [44], there is a positive relationship between national income (GDP) and economic welfare; the relationship is not linear, and the impact of GDP on welfare diminishes beyond a certain threshold. They also argued that this may be due to issues such as income inequality, environmental degradation, and social disparities that traditional GDP measures may not fully capture.

Another study by Al-shami, Al Mamun [45] explored the relationship between national income accounting and economic welfare in Pakistan’s environmental sustainability context. They used the Genuine Progress Indicator (GPI), an alternative measure of economic welfare that adjusts GDP for environmental and social factors, to assess economic welfare in Pakistan. The findings revealed that while GDP has been growing in Pakistan, the GPI, which accounts for environmental costs, has declined, indicating that economic growth may not necessarily translate into sustainable economic welfare. Furthermore, subjective well-being and happiness have been increasingly recognized as important indicators of economic welfare.

Shahzad and Siddiqui (2018) examined the relationship between subjective well-being and income in Pakistan. They found that while income positively impacts emotional well-being, other factors such as education, health, and social support are also significantly determined. This suggests that a broader perspective of economic welfare that includes subjective well-being can provide valuable insights into the well-being of individuals and communities in Pakistan.

Overall, the literature on national income accounting and economic welfare in Pakistan suggests that GDP may not fully capture the multidimensional aspects of economic welfare, including income inequality, environmental sustainability, and subjective well-being. Alternative measures such as the GPI and subjective well-being indicators can provide a more comprehensive assessment of economic welfare in Pakistan. Further research and policy discussions are needed to understand better the relationship between national income accounting and economic welfare in Pakistan and to develop policies that promote sustainable and inclusive economic welfare in the country. On the ground of the previous theory and literature background, we developed the following hypothesis,

***H1*:** Savings in the country have a significant positive impact on Pakistan’s economic welfare.
***H2*:** GDP per capita has a significant positive impact on economic welfare.
***H3*:** Foreign direct investment outflow significantly negatively impacts economic welfare.
***H4*:** The GDP growth rate has a significant positive impact on Pakistan’s economic welfare.
***H5*:** Total market capitalizations of the firms have a negative impact on the economic welfare.
***H6*:** Pakistan’s trade flow with other nations has a significant positive impact on economic welfare.
***H7*:** Lending interest rate has a significant negative impact on economic welfare.
***H8*:** The inflation rate has a significant negative impact on economic welfare.
***H9*:** Population growth has a negative impact on economic welfare.

Fig 2 represents the study’s conceptual framework that provides our research roadmap for investigating our research objectives.

**Fig 2:** Conceptual framework.

## Material and methods

To meet the study’s objective, we collected data on the national accounting of different parameters and economic welfare factors from the World Bank data portal annually for emerging economies such as Pakistan from 1950 to 2022. From the emerging economies, Pakistan was selected based on the volatility in the growth rate due to some political, economic, and social factors, and data is available due to the coordination of the international monetary and health organizations that work in Pakistan. Another reason for selecting Pakistan from the merging economy is that there is a lack of economic welfare due to the scarcity of resources as the unemployment rate is high, about 6.42 percent, and it has an increasing trend. Moreover, life expectancy and age dependency are decreasing due to the lack of health facilities in Pakistan. Many United Nations welfare organizations work for the economic welfare of Pakistan, which provides further evidence of the sufficiency of economic welfare. A wide range of data is selected based on the different democratic regime changes in Pakistan, and every government has the task of working for economic welfare. Still, they cannot obtain their target due to the lack of facilities and other policymaking. Moreover, Table 1 represents the measurement of the independent variables, and Table 2 represents the measurement of the dependent variables.

**Table 1:** Measurement of independent variable.

*independent variable*	*Sign*	*Measurement*	*Reference*
Savings	SAV	Gross domestic savings (% of GDP)	World Bank national accounts data, and OECD National Accounts data files.
GDP per capita	GDPC	GDP per capita (constant 2015 US$)	World Bank national accounts data, and OECD National Accounts data files.
FDI	FDI	Foreign direct investment, net inflows (% of GDP)	International Monetary Fund, International Financial Statistics and Balance of Payments databases, World Bank, International Debt Statistics, and World Bank and OECD GDP estimates.
GDP Growth	GDP	GDP per capita growth (annual %)	World Bank national accounts data, and OECD National Accounts data files.
Market capitalization	MC	The market capitalization of listed domestic companies (% of GDP)	World Federation of Exchanges database.
Trade	TRA	Trade (% of GDP)	World Bank national accounts data, and OECD National Accounts data files.
Inflation	INF	Inflation, consumer prices (annual %)	International Monetary Fund, International Financial Statistics, and data files.
Population growth	PGR	Population growth (annual %)	It was derived from the total population. Population source: (1) United Nations Population Division. World Population Prospects: 2022 Revision, (2) Census reports and other statistical publications from national statistical offices, (3) Eurostat: Demographic Statistics, (4) United Nations Statistical Division. Population and Vital Statistics Report (various years), (5) U.S. Census Bureau: International Database, and Secretariat of the Pacific Community: Statistics and Demography Program.
Lending interest rate	LINT	Lending interest rate (%)	International Monetary Fund, International Financial Statistics, and data files.

Authors sources

**Table 2:** Measurement of dependent variables.

Dependent variable	Sign	Measurement	Reference
Unemployment	UNP	Youth unemployment refers to the share of the labor force ages 15–24 without work but available for and seeking employment. Definitions of labor force and unemployment differ by country.	World Bank data portal
Life expectancy	LIFE	Life expectancy at birth indicates the number of years a newborn infant would live if prevailing patterns of mortality at the time of its birth were to stay the same throughout its life.	World Bank data portal
Age dependency ratio	ADR	The age dependency ratio, young (% of working-age population)	World Bank data portal
legal right	L.R.	Strength of legal rights index (0 = weak to 12 = strong)	World Bank data portal
Mortality rate C	MRC	Mortality rate under 5 (per 1,000 live births)	World Bank data portal

The econometric model of the study is given below,

$$\begin{array}{l} UNP_{\mathrm{it}}=\alpha_{0}+\beta_{1}{\left(SAV\right)}_{\mathrm{it}}+\beta_{2}{\left(GDP\right)}_{\mathrm{it}}+\beta_{3}{\left(GDPC\right)}_{\mathrm{it}}+\beta_{4}{\left(FDI\right)}_{\mathrm{it}}+\beta_{5}{\left(MC\right)}_{\mathrm{it}}+\beta_{6}{\left(TRA\right)}_{\mathrm{it}}+\\ \beta_{7}{\left(INF\right)}_{\mathrm{it}}+\beta_{8}{\left(PGR\right)}_{\mathrm{it}}+\beta_{9}{\left(LINT\right)}_{\mathrm{it}}+\varepsilon_{\mathrm{it}} \end{array}$$

$$\begin{array}{l} LIFE_{\mathrm{it}}=\alpha_{0}+\beta_{1}{\left(SAV\right)}_{\mathrm{it}}+\beta_{2}{\left(GDP\right)}_{\mathrm{it}}+\beta_{3}{\left(GDPC\right)}_{\mathrm{it}}+\beta_{4}{\left(FDI\right)}_{\mathrm{it}}+\beta_{5}{\left(MC\right)}_{\mathrm{it}}+\beta_{6}{\left(TRA\right)}_{\mathrm{it}}+\\ \beta_{7}{\left(INF\right)}_{\mathrm{it}}+\beta_{8}{\left(PGR\right)}_{\mathrm{it}}+\beta_{9}{\left(LINT\right)}_{\mathrm{it}}+\varepsilon_{\mathrm{it}} \end{array}$$

$$\begin{array}{l} ADR_{\mathrm{it}}=\alpha_{0}+\beta_{1}{\left(SAV\right)}_{\mathrm{it}}+\beta_{2}{\left(GDP\right)}_{\mathrm{it}}+\beta_{3}{\left(GDPC\right)}_{\mathrm{it}}+\beta_{4}{\left(FDI\right)}_{\mathrm{it}}+\beta_{5}{\left(MC\right)}_{\mathrm{it}}+\beta_{6}{\left(TRA\right)}_{\mathrm{it}}+\\ \beta_{7}{\left(INF\right)}_{\mathrm{it}}+\beta_{8}{\left(PGR\right)}_{\mathrm{it}}+\beta_{9}{\left(LINT\right)}_{\mathrm{it}}+\varepsilon_{\mathrm{it}} \end{array}$$

$$\begin{array}{l} LR_{\mathrm{it}}=\alpha_{0}+\beta_{1}{\left(SAV\right)}_{\mathrm{it}}+\beta_{2}{\left(GDP\right)}_{\mathrm{it}}+\beta_{3}{\left(GDPC\right)}_{\mathrm{it}}+\beta_{4}{\left(FDI\right)}_{\mathrm{it}}+\beta_{5}{\left(MC\right)}_{\mathrm{it}}+\beta_{6}{\left(TRA\right)}_{\mathrm{it}}+\\ \beta_{7}{\left(INF\right)}_{\mathrm{it}}+\beta_{8}{\left(PGR\right)}_{\mathrm{it}}+\beta_{9}{\left(LINT\right)}_{\mathrm{it}}+\varepsilon_{\mathrm{it}} \end{array}$$

$$\begin{array}{l} MRC_{\mathrm{it}}=\alpha_{0}+\beta_{1}{\left(SAV\right)}_{\mathrm{it}}+\beta_{2}{\left(GDP\right)}_{\mathrm{it}}+\beta_{3}{\left(GDPC\right)}_{\mathrm{it}}+\beta_{4}{\left(FDI\right)}_{\mathrm{it}}+\beta_{5}{\left(MC\right)}_{\mathrm{it}}+\beta_{6}{\left(TRA\right)}_{\mathrm{it}}+\\ \beta_{7}{\left(INF\right)}_{\mathrm{it}}+\beta_{8}{\left(PGR\right)}_{\mathrm{it}}+\beta_{9}{\left(LINT\right)}_{\mathrm{it}}+\varepsilon_{\mathrm{it}} \end{array}$$

The Ordinary Least Squares (OLS) method is a popular statistical technique used in business analysis to estimate the relationship between a dependent variable and one or more independent variables. OLS is commonly used in regression analysis to identify the strength and direction of the relationship between variables (Mohammed et al., 2021), and another study used OLS regression analysis to examine the relationship between ethical leadership and employee well-being [46]. Moreover, the OLS method has been widely used in business analysis to investigate various relationships and inform decision-making. Its versatility and ease of use have made it a popular technique among researchers and practitioners.

Numerous studies have highlighted the usefulness of regression analysis in various fields, including finance, economics, and medicine. One recent study examined the relationship between economic growth and foreign direct investment (FDI) in the ASEAN region. The researchers used multiple regression analysis to analyze the data [47]. Another used regression analysis to examine the relationship between China’s stock market returns and exchange rates [48]. In medicine, a study used regression analysis to analyze patient satisfaction with healthcare services [49].

The Generalized Method of Moments (GMM) is used as the robustness analysis in this study to make more effective results that should be valuable for conclusions. Moreover, there is an increasing trend of simultaneous effects between the variables for various reasons. The regression analysis is insufficient to diagnose the simultaneous effect simultaneously; that’s why the GMM captures the simultaneous effects and improves the findings by providing real impact and relationship between exogenous and endogenous variables.

GMM is a widely used econometric technique for estimating parameters in various economic and financial models. Its effectiveness has been extensively discussed and examined in previous literature. GMM’s efficiency and consistency in estimating parameters, particularly in the presence of endogeneity, measurement error, or other forms of model misspecification, is one of its primary strengths. Several studies, including those by Hansen (1982) and Arellano and Bond (1991), illustrate this model specification. GMM is a versatile method that may analyze various economic models. Researchers have used GMM to estimate parameters in models relating to macroeconomics, finance, labor economics, and other fields. This adaptability is mentioned by Newey and McFadden (1994).

Moreover, we decided to use the method of estimation GMM to analyze time series data because of its flexibility, efficiency, and capacity to handle complicated data structures [50]. GMM in time series analysis allows researchers to address endogeneity, non-stationarity, and serial correlation by establishing moment conditions based on the data-generating process [51]. By employing instrumental variables and accepting diverse transformations, GMM allows consistent parameter estimates while relaxing strict distributional assumptions [52]. Moreover, GMM can minimize the simultaneous effect in the model [53], and that’s why we used GMM as the estimation method in our study for robustness analysis in time series data.

## Findings and discussions

Table 3 shows the descriptive statistics. The descriptive statistics show that the age dependency ratio is 77.13 for Pakistan, with a maximum value of 85 and a minimum value of 62.78. The FDI has a mean value of 0.6161, with a maximum of 3.688 and a minimum of 0.062. The GDP growth rate average of the selected period for Pakistan is 2.27%, with a maximum of 8.32%. The per capita income of the nation is an average of 861 annually.

**Table 3:** Descriptive statistics.

	Mean	Median	Maximum	Minimum	skewness	kurtosis	Std. Dev.
UNP	2.633	0.000	13.410	0.000	-0.0198	2.3493	4.184
ADR	77.136	79.404	85.452	62.782	-0.0182	2.1429	6.585
LR	0.226	0.000	2.000	0.000	0.0912	3.809	0.638
LIFE	11.035	10.758	16.785	7.347	0.0204	3.1067	1.797
MRC	139.526	138.450	251.900	63.300	-0.0121	1.727	50.452
SAV	11.180	11.197	17.399	5.376	-0.3211	3.0866	3.512
GDPC	861.629	869.840	1473.865	371.063	0.1241	1.833	303.269
FDI	0.616	0.480	3.668	-0.063	-0.0432	2.761	0.746
GDP	2.275	2.158	8.322	-2.970	0.01651	1.1429	2.291
MC	5.872	0.000	45.749	0.000	-0.0413	3.7614	11.403
TRA	29.415	31.112	38.499	15.821	0.0551	3.6721	5.918
LINT	3.219	0.000	14.538	0.000	-0.0771	1.8741	5.217
INF	8.040	7.209	26.663	-0.516	-0.1132	3.0876	5.137
PGR	2.607	2.648	4.423	0.000	0.1412	2.871	0.781

Moreover, inflation has a mean value of 8% in the economy, but legal right has an average value of 0.22. The lending interest rate remains at an average of 3.12%, with a maximum of 14%. However, market capitalization averages 5.87, and the mortality rate in Children averages 139.52. Saving has a mean value of 11.86%, but the trade has 29% of the total market capitalization. Table 4 shows that all the correlation values between variables are less than 0.80, except for the mortality rate in children and the GDP per capita, indicating a low correlation between them.

**Table 4:** Correlation matrix.

	ADR	FDI	GDP	GDPC	INF	LIFE	LINT	LE	MC	MR	PGR	SAV	TRA	UNP
ADR	1													
FDI	-0.26	1												
GDP	-0.062	-0.139	1											
GDPC	-0.664	0.545	-0.151	1										
INF	0.12	0.216	-0.24	0.103	1									
LR	-0.604	0.027	0.139	0.559	-0.154	1								
LINT	-0.705	0.552	-0.08	0.769	0.173	0.483	1							
LIFE	-0.027	0.326	-0.223	0.334	0.079	0.308	0.276	1						
MC	-0.039	0.749	-0.106	0.317	0.178	-0.185	0.372	0.254	1					
MR	0.545	-0.572	0.203	-0.974	-0.144	-0.467	-0.717	-0.418	-0.371	1				
PGR	0.726	-0.205	0.026	-0.433	0.112	-0.548	-0.613	0.002	-0.112	0.31	1			
SAV	0.546	0.146	-0.024	-0.112	-0.069	-0.36	-0.366	0.169	0.36	-0.002	0.235	1		
TRA	0.131	0.456	-0.162	0.403	0.466	-0.063	0.153	0.374	0.354	-0.481	0.321	0.105	1	
UNP	-0.044	0.157	-0.111	0.428	0.034	0.19	0.086	0.008	0.198	-0.437	-0.114	0.359	0.245	1

Author Source.

In Table 5, our regression results show that foreign direct investment outflow, Gross domestic product growth rate, GDP per capita, higher Interest, market capitalization, and population growth have significant negative. In contrast, trade and savings significantly positively impact the unemployment rate. Moreover, all the factors of the national income accounting have a significant positive relationship with Life expectancy, which means that when the national income factors increase, the economic welfare Life expectancy increases due to better health facilities, many resources, and correct economic policies. However, foreign direct investment, inflation rate, lending interest rate, and population growth have significant positive, while GDP growth, GDP per capita, and the interest rate have a negative impact on age dependency. Similarly, all the national income accounting factors decrease the legal rights within the economy due to a significant negative relationship. Moreover, there is a negative significant relationship between national income accounting attributes and motility rate within the children.

**Table 5:** Results of regression.

	UNP	LIFE	ADR	LR	MR
Independent variable	Coefficient (P)	Coefficient (P)	Coefficient (P)	Coefficient (P)	Coefficient (P)
FDI	-1.051** (0.021)	0.059** (0.020)	0.752** (0.014)	-0.176* (0.062)	0.789 (0.702)
GDP	-0.105** (0.0597)	0.087 (0.387)	-0.176 (0.104)	0.073*** (0.001)	0.904* (0.065)
GDPC	-0.010*** (0.001)	0.124** (0.021)	-0.006*** (0.001)	0.002*** (0.000)	-0.159*** (0.000)
INF	0.023 (0.822)	0.001** (0.051)	0.210*** (0.001)	0.002 (0.889)	-0.084 (0.737)
MC	-0.224** (0.0249)	0.009 (0.753)	-0.703*** (0.000)	-0.053** (0.015)	-0.805* (0.091)
LINT	-0.109** (0.049)	1.000*** (0.000)	0.063** (0.059)	0.029*** (0.000)	-0.266** (0.048)
PGR	-0.846** (0.031)	0.097 (0.355)	1.618*** (0.002)	-0.329*** (0.001)	-8.110*** (0.000)
SAV	0.511*** (0.002)	1.970*** (0.006)	0.455*** (0.000)	-0.065*** (0.000)	-1.455*** (0.000)
TRA	0.108** (0.0382)	3.978*** (0.000)	0.083 (0.268)	-0.017 (0.199)	-0.076 (0.800)

Note. Results are significant at 1%, 5%, and 10% significance levels, indicating

***, **, and *, respectively.

According to Humpe and Macmillan [54], Malik [55], cointegration analysis is the best technique for modelling the relationship and is also helpful in testing the simultaneous effect found between the selected variables. All the variables were first difference stationery. After the stationarity, we try the cointegration pattern between selected variables. All the values were significant and indicated that the cointegration is found between the variables, and the previous method, such as the regression analysis, is not helpful due to the simultaneous effect found between the selected variables. Our preliminary test of the cointegration successfully validated our findings of the GMM method.

The GMM method is helpful to remove the simultaneous effect. When cointegration between variables is found, it shows the simultaneous effect available between the selected variables. In our analysis, all variables are coined and show the simultaneous effect is found between them. The results of the cointegration are shown in Table 6.

**Table 6:** Cointegration test.

Johansen normalized cointegrating results.										
	UNP		LIFE		ADR		LR		MR	
	Coef.	Z	Coef.	Z	Coef.	Z	Coef.	Z	Coef.	Z
FDI	-0.143***	-82.19	0.873***	28.29	-0.871***	-78.23	-0.981***	-72.19	0.222***	78.99
GDP	-0.152***	-92.23	0.872***	28.98	-0.561***	-78.19	-0.871***	-82.23	0.531	72.98
GDPC	0.124***	34.87	0.541***	56.87	0.528***	23.87	0.542	64.87	0.128	34.87
INF	-0.521***	-18.90	-0.249***	-34.12	-0.361	-19.80	-0.541	-19.00	0.651***	18.90
MC	0.614***	18.17	0.241***	22.98	0.871***	17.17	0.881***	19.17	0.552***	18.17
LINT	-0.152***	-37.74	0.651***	26.87	-0.451	-87.87	-0.152***	-37.74	-0.651***	-37.87
PGR	0.515***	54.57	0.125***	34.76	0.718**	44.57	0.515*	76.57	0.515	74.44
SAV	-0.187***	-34.87	0.761***	20.76	-0.281***	-53.87	-0.187**	-34.87	-0.189	-34.74
TRA	0.615***	18.90	0.261***	19.91	0.871***	34.94	0.691***	18.99	0.223***	21.14

Note: Results are significant at 1%,5%, and 10% significance levels and represented by

***, **, and *, respectively.

The GMM findings are shown in Table 7, used as a robustness analysis of the regression method. Our findings demonstrate the high strength in the coefficient with the same direction as found by the regression, but GMM findings are more improved with the improvement in the relation due to increasing the strength of the coefficient. From the GMM method, we find out that the previous value of unemployment also affects the current employment rate by 0.043. Moreover, the last value of the Life expectancy also contributed to the existing value by 0.001. The previous value of the age dependency is also helpful in predicting the current value by 0.002. The last value of the legal rights and mortality rate also affects the current value by 0.001 and 0.006, respectively.

**Table 7:** Robustness analysis: Generalized method of movement (GMM).

	UNP	LIFE	ADR	LR	MR
Independent	Coefficient (P)	Coefficient (P)	Coefficient (P)	Coefficient (P)	Coefficient (P)
UNP (-1)	0.043 (0.000)	-	-	-	-
LIFE (-1)	-	0.001 (0.000)	-	-	-
ADR (-1)	-	-	0.002 (0.000)	-	-
LR (-1)	-	-	-	0.001 (0.000)	-
MR (-1)	-	-	-	-	0.006 (0.000)
FDI	-1.091 (0.001)	0.086 (0.000)	0.971 (0.002)	-0.342 (0.001)	0.672 (0.514)
GDP	-0.309 (0.008)	0.096 (0.564)	-0.321 (0.209)	0.132 (0.000)	0.805 (0.004)
GDPC	-0.070 (0.000)	0.324 (0.000)	-0.015 (0.000)	0.012 (0.000)	-0.320 (0.000)
INF	0.043 (0.822)	0.051 (0.000)	0.210 (0.000)	0.122 (0.978)	-0.076 (0.564)
MC	-0.432 (0.000)	0.023 (0.532)	-0.709 (0.000)	-0.076 (0.000)	-0.902 (0.000)
LINT	-0.109 (0.000)	1.043 (0.000)	0.072 (0.000)	0.124 (0.000)	-0.896 (0.000)
PGR	-0.971 (0.000)	0.176 (0.671)	1.871 (0.000)	-0.432 (0.000)	-7.751 (0.000)
SAV	0.689 (0.000)	1.991 (0.000)	0.541 (0.000)	-0.192 (0.000)	-1.561 (0.000)
TRA	0.381 (0.000)	3.231 (0.000)	0.102 (0.162)	-0.209 (0.281)	-0.190 (0.311)

Note: Results are significant at 1%,5%, and 10% significance levels.

Moreover, foreign direct investment outflows, GDP growth rates, GDP per capita, higher interest rates, market capitalization, and population growth have a significant negative impact on the unemployment rate, with a more pronounced effect when compared to regression analysis results. Conversely, trade and savings have a significant positive effect on the unemployment rate.

Furthermore, all national income accounting parameters substantially relate to life expectancy. In our Generalized Method of Moments (GMM) analysis, however, foreign direct investment, the inflation rate, loan interest rates, and population growth have a significant positive impact on age dependency, but GDP growth, GDP per capita, and interest rates have a negative effect. Notably, the magnitude of these impacts corresponds to the findings of our regression study.

Similarly, all components in national income accounting contribute to a decline in legal rights inside the economy due to a significant negative link. Furthermore, a substantial negative association between national income accounting features and child mortality rates is revealed.

Based on our results utilizing the GMM method, we can conclude that this method enhanced the coefficients and significance level. However, it has not changed the direction of these impacts, demonstrating the correctness of our estimation method. As a result, we rely on the GMM technique results to reach our conclusions because they are more accurate and reliable.

## Discussion of findings

From our results, we find that FDI outflow has a significant negative impact on the unemployment rate. It means that when the FDI outflow increases, the unemployment within the economy decreases, leading to a decrease in the economic welfare within Pakistan. On the other hand, when FDI inflow increases, then unemployment within the country decreases. In this way, our findings are consistent with the findings of Chang [56], who found a positive linkage between FDI and the unemployment rate. He also concluded that the employment rate rises from the FDI, which generates business opportunities within the economy and leads to skilled and unskilled employees.

Gross domestic product and GDP per capita have a significant negative impact on the unemployment rate, indicating that when the GDP increases, the employment rate within the economy increases due to an increase in the production, manufacturing, and trading of the goods that produce the employment opportunities. Consistent with the Keynesian theory that suggests an increase in GDP can lead to higher employment through the concept of aggregate demand. Moreover, increased demand for goods and services leads to increased production, which requires businesses to hire more workers, resulting in employment growth. When the economy is operating below its potential GDP, government intervention through fiscal policy, such as increased government spending or tax cuts, can stimulate aggregate demand and lead to higher GDP and employment. In this way, Keynesian theory has the same remarks as we discussed, for rising GDP creates employment opportunities by expanding business concerns that lead to economic welfare.

In our findings, lending interest rate has a significant negative impact on Pakistan’s unemployment rate. The higher lending interest rates can lead to reduced borrowing by businesses and individuals, potentially limiting economic activity and job creation, thereby contributing to higher unemployment [57]. Our findings are similar to those of Bhutta and Keys [57]. Moreover, these findings align with the credit channel theory, which suggests that fluctuations in interest rates can affect the availability of credit and employment. Conversely, some studies argue that central banks may implement higher interest rates to combat inflation, and lower inflation can positively impact job stability and the unemployment rate, as it fosters economic confidence and investment. The impact of lending interest rates on unemployment is thus contingent on various economic conditions and policy objectives, making it a complex and multifaceted relationship that requires careful consideration. Moreover, the inflation rate has no significant findings in our analysis in either regression or GMM estimation methods.

Trade and saving have a positive impact on unemployment because in Pakistan, due to the diverse policy of the government recently, the rich have become rich, and poor people face many troubles due to hoarding and other reasons. Our findings reject the null hypothesis and accept the alternative hypothesis that the foreign direct investment outflow from the country leads to an increase in the unemployment rate within the economy. In this way, our findings are opposite to Nwaka, Uma, and Tuna’s (2015) conclusions that trade increases the employment rate in the nation by providing different opportunities to business openers. Similarly, our findings are similar to the Dix-Carneiro, Pessoa [58] that concluded the mobilization of savings to generate income and increase the employment rate in the emerging economy. In the emerging economy, rich people do not mobilize their savings but hold them for some purposes with negative consequences.

Moreover, the results show that the GDP and GDP per capita lead to decreased unemployment and increased economic welfare within the nation. A growing GDP signifies a larger economy with more economic activity and job opportunities, which, in turn, can help reduce unemployment. Additionally, as GDP per capita rises, it generally implies an improved standard of living and greater individual purchasing power. This can lead to higher demand for goods and services, further stimulating economic growth and job creation. Moreover, a higher GDP per capita is often associated with improved public infrastructure, education, and healthcare, which can enhance the population’s overall well-being. However, the effectiveness of this relationship also depends on the distribution of wealth and access to opportunities within society, as an unequal distribution can hinder the positive impacts on unemployment reduction and overall economic welfare. Similarly, our findings are supported by the previous study findings of Henares Montiel, Ruiz Pérez [59].

However, all the factors of the national income accounting have a significant positive relationship with Life expectancy, and it means that when the national income factors increase, the economic welfare Life expectancy increases due to better health facilities, many resources, and correct economic policies. In this way, our findings are consistent with the previous findings of Nordhaus [60], who concluded the same findings. In this way, our null hypothesis was rejected with the justification that the national accounting attributes higher value to increase the economic welfare through expanding the life expectancy within Pakistan.

Moreover, results show that GDP, GDP per capita, and the interest rate significantly negatively impact age dependency. The link between GDP, GDP per capita, and interest rates is complicated by age dependency. Higher GDP and GDP per capita generally indicate a more prosperous economy, which can provide a higher standard of living for the working-age population and improved access to healthcare and social services, reducing age dependency as older people may be less economically dependent. However, lower birth rates in more economically developed countries may negatively impact age dependency, leading to an aging population [61].

Conversely, the interest rate can influence age dependency through its impact on savings and investment. High interest rates can encourage savings and investment, potentially leading to more financial security for older individuals and reducing age dependency [62]. In this way, our findings are similar to Lusardi, Mitchell [62]. Nonetheless, the relationship between these economic factors and age dependency is influenced by various demographic, cultural, and policy-related factors, making it essential to consider the broader context when assessing their effects on age dependency.

When these factors increase, then age dependency decreases because it is a multifaceted issue that involves not only economic factors but also social, cultural, and demographic aspects. Therefore, it’s crucial to carefully analyze and consider the specific circumstances and dynamics when examining the relationship between these factors and age dependency. Foreign direct investment, savings, and trade increase Age dependency because the results are significant and positive. In this way, our findings are consistent with the previous findings of Aibai, Huang [63].

However, most of the national income accounting attributes are significant and negative regarding legal rights in Pakistan, which means that all the national income accounting factors decrease the legal rights within the economy. In this way, our findings are opposite to those of Zhou, Xiao, and Yao (2010), who concluded that national income accounting factors indirectly influence economic legal rights. The relationship is complex and multifaceted. For example, a higher GDP or GDP per capita may indicate economic growth and potentially increased resources for the government to invest in legal infrastructure, such as the judiciary, law enforcement agencies, and regulatory institutions, which can enhance legal rights. Additionally, interest rates, which are set by monetary authorities, impact borrowing costs, investments, and overall economic activity, which can indirectly affect legal rights related to business contracts and investments.

However, the results are significant and show a negative relationship between national income accounting and the mortality rate of children. It means that when there is prosperity within the economy, all the children are safe, fully nutritious, and healthy. In this way, our findings are consistent with the previous findings of Preston [64], who concluded that prosperity increases children’s health and leads to decreased mortality. One of the main reasons for this negative relationship is that higher national income accounting measures generally indicate more significant economic development and improved living standards, which positively affect children’s health and well-being.

Higher national income accounting measures are often associated with increased access to healthcare facilities, including maternal and child healthcare services. This can lead to improved prenatal care, nutrition, vaccination coverage, and overall healthcare for children, which can help reduce child mortality rates. These factors are also linked to improved nutrition and food security, as increased income levels allow for better access to nutritious food. Malnutrition is a significant risk factor for child mortality, and improved nutrition helps reduce the risk of child deaths due to malnutrition-related causes. These factors of the national accountings are often associated with improved access to safe water and sanitation facilities, which can contribute to better hygiene practices and reduce the risk of waterborne diseases. Access to clean water and sanitation facilities can directly impact child health and mortality rates.

However, the higher national income accounting measures are often linked to increased access to education, including maternal education. Maternal education is associated with better knowledge and practices related to child health and care, which can impact child mortality rates. The national income accounting attributes are generally associated with improved socio-economic development, including poverty reduction, improved infrastructure, and social protection programs. These factors contribute to better living conditions and reduced vulnerability, impacting child mortality rates. Moreover, Table 8 represents the hypothesis decision.

**Table 8:** Decision of the hypothesis.

Hypothesis Statement	Decision of alternative	Reason
***H1*:** Savings in the country have a significant positive impact on Pakistan’s economic welfare.	Accept	Saving significant with all proxies of economic welfare
***H2*:** GDP per capita has a significant positive impact on economic welfare.	Partial Accept	All are significant, but with life expectancy, they are not substantial.
***H3*:** Foreign direct investment outflow significantly negatively impacts economic welfare.	Partial Accept	All are significant, but the mortality rate for children is not significant.
***H4*:** The GDP growth rate has a significant positive impact on Pakistan’s economic welfare.	Accept	GDP is significant with all proxies of economic welfare
***H5*:** Total market capitalizations of the firms have a negative impact on the economic welfare.	Partial Accept	All are significant, but with life expectancy, they are not significant.
***H6*:** Pakistan’s trade flow with other nations has a significant positive impact on economic welfare.	Partial Accept	Relationship with age dependency, legal right, and mortality rate children not significant.
***H7*:** Lending interest rate has a significant negative impact on economic welfare.	Accept	Interest rate significant with all proxies of economic welfare
***H8*:** The inflation rate has a significant negative impact on economic welfare.	Partial Accept	The relationship between unemployment, legal rights, and children’s mortality rate is insignificant.
***H9*:** Population growth has a negative impact on economic welfare.	Partial Accept	Relationship with life expectancy not significant

Author Source

## Conclusion and recommendations

In conclusion, every economy is responsible for providing economic welfare to its citizens. The accounting attributes such as GDP, interest rate, market capitalization, and high population growth decrease the unemployment rate in Pakistan. When these factors increase, business opportunities within the country lead to employment of the number of populations in the business concern. Moreover, an increase in the national income accounting attributes leads to a rise in Life expectancy, which means that when the national income factors increase, then the factor of the economic welfare Life expectancy increases due to the better health facilities, many resources, and correct economic policies.

Similarly, a rise in the national income accounting attributes such as foreign direct investment, inflation rate, lending interest rate, and population growth leads to a rise in age dependency. An increase in foreign direct investment and population growth may boost economic activity. However, suppose this growth is not balanced by sufficient job creation and economic opportunities. In that case, it can lead to a higher dependency ratio, as a larger working-age population must support more dependents. High inflation and lending interest rates can affect retirees’ purchasing power and make it challenging for older people, contributing to age dependency.

Moreover, higher GDP growth often implies increased economic opportunities, reducing age dependency as more people can support dependents. Additionally, higher GDP per capita indicates improved living standards, potentially resulting in better support for elderly populations. These factors can collectively mitigate age dependency.

When mismanaged, national income accounting factors like GDP growth, inflation, and interest rates can divert resources and attention from protecting legal rights. Poor economic conditions may reduce government resources for legal infrastructure, potentially eroding legal rights enforcement. However, the impact on legal rights depends on a given country’s specific policies and governance.

Moreover, the higher national income accounting measures are generally associated with improved child health and well-being, including better access to healthcare, improved nutrition and food security, better water and sanitation facilities, increased education, and overall socio-economic development. These factors contributed to reducing child mortality rates by addressing various risk factors and improving general living conditions. However, it’s important to note that the relationship between national income accounting factors and child mortality rates is complex and is influenced by multiple factors. Government policies, healthcare systems, social and cultural norms, and demographic factors also play a role in determining child mortality rates.

Overall, the findings highlight the importance of economic development and improved living standards in reducing child mortality rates, increasing the unemployment rate, and increasing life expectancy. Policies and interventions that strengthen national income accounting measures and address other social and healthcare-related factors can positively impact child health and well-being, lowering child mortality rates. Further research and evidence-based policies are needed to understand better the complex relationship between national income accounting factors and child mortality rates and effectively address this critical public health issue.

The study has several important implications for policymakers, practitioners, and other stakeholders. The policymakers design and implement policies that promote economic growth and improve welfare outcomes within the economy. By measuring the distribution of income and wealth across different groups in society, policymakers can design more targeted policies that address income inequality and promote inclusive growth. National income accounting provides a framework for measuring the overall economic performance of a country and forecasting future economic growth. Moreover, policymakers make more informed decisions about financial planning and resource allocation. This study also has significant implications for providing a common framework for comparing the economic performance of different countries. However, using the study’s findings, policymakers can identify best practices and policies that can be adapted to their own country’s context and nature.

This study also provides significant implications for businesses and investors by providing new evidence about the economic welfare distribution within Pakistan. By using the information, investors invest in a well-organized nation that contributes to economic welfare; in this way, investors get confidence in the economic indicator of the respected economy. Moreover, the existing businesses’ concerns can help make more informed decisions about investment and expansion opportunities. Ultimately, the study has important implications for social welfare outcomes that increase the value of their stakeholders, such as the population. By improving economic performance and promoting inclusive growth, policymakers can improve citizens’ quality of life and promote social welfare outcomes such as health, education, and employment.

This study has some limitations and provides a road map for future research topics for investigations. Initially, it relies heavily on standard national income accounting measurements such as GDP, savings, and investment, which may not fully depict a population’s economic well-being, particularly in emerging nations with extensive informal sectors. Second, it may neglect the distributional features of economic well-being, which are critical in understanding inequality and poverty. Future research in this field should look into more nuanced and inclusive metrics of economic well-being that consider income inequality, access to critical services, environmental sustainability, and the unique difficulties and dynamics of rising countries. Furthermore, combining contemporary data analytics and approaches can provide more precise and real-time knowledge of the relationship between national income accounting features and economic welfare in these circumstances. Future studies must investigate more holistic indicators that better reflect the complex socio-economic dynamics of rising economies. Researchers should create complete frameworks that include money, health, education, career prospects, and environmental sustainability to provide a more nuanced view of economic well-being. Similarly, future research should be conducted on economic welfare, such as health factors, educational factors, and environmental protection factors as economic welfare.

The influence of policy interventions and structural reforms should be taken as moderating variables between national income accounting and economic welfare in future topics. Using contemporary data analytics and advanced econometric methodologies can improve the accuracy and timeliness of data collection and analysis, creating more informed policies and plans for attaining sustainable and inclusive economic growth in these situations. Therefore, more accurate and comprehensive data and data analysis techniques, such as the wavelet approach, should be used in future research. Due to limitations, this study comprises Pakistan, but future research may investigate the multi-country and cross comparison of these economies in different contexts.
